The article "Relationship between epithelial-to-mesenchymal transition and the inflammatory microenvironment of hepatocellular carcinoma" was published in 2018. Journal: J Exp Clin Cancer Res.

# Relationship between epithelial-to-mesenchymal transition and the inflammatory microenvironment of hepatocellular carcinoma

**DOI:** 10.1186/s13046-018-0887-z

**Published:** 2018-08-29

**Authors:** Long Yan, Feng Xu, Chao-liu Dai

**Affiliations:** Department of Hepatobiliary and Splenic Surgery, Sheng Jing Hospital of China Medical University, No.36 Sanhao Street, Heping District, Shenyang, Liaoning China

**Keywords:** Hepatocellular carcinoma, Epithelial-to-mesenchymal transition, Inflammatory microenvironment, Tumor-related macrophages, Expressed products of infected virus

## Abstract

Epithelial-to-mesenchymal transition (EMT) is a complex process involving multiple genes, steps and stages. It refers to the disruption of tight intercellular junctions among epithelial cells under specific conditions, resulting in loss of the original polarity, order and consistency of the cells. Following EMT, the cells show interstitial cell characteristics with the capacity for adhesion and migration, while apoptosis is inhibited. This process is critically involved in embryogenesis, wound-healing, tumor invasion and metastasis. The tumor microenvironment is composed of infiltrating inflammatory cells, stromal cells and the active medium secreted by interstitial cells. Most patients with hepatocellular carcinoma (HCC) have a history of hepatitis virus infection. In such cases, major components of the tumor microenvironment include inflammatory cells, inflammatory factors and virus-encoded protein are major components. Here, we review the relationship between EMT and the inflammatory tumor microenvironment in the context of HCC. We also further elaborate the significant influence of infiltrating inflammatory cells and inflammatory mediators as well as the products expressed by the infecting virus in the tumor microenvironment on the EMT process.

## Background

Hepatocellular carcinoma (HCC) is one of the most common malignant tumors worldwide and is a typical inflammatory-related tumor that is associated with early metastasis and poor prognosis. From a global perspective, between 75 and 80% of patients with liver cancer have a history of chronic hepatitis B virus (HBV) and hepatitis C virus (HCV) infections [1, 2]. Sub-Saharan Africa and East Asia are regions with a high incidence of hepatocellular carcinoma, and the HCC patients in China account for 50% of the total number of patients around the world, a fact that is inseparable from the huge numbers of people with hepatitis infections in this region [3]. In addition, the accumulation of toxic compounds (such as alcohol and aflatoxins) as well as metabolic liver injury are also important causative factors in the development of liver cancer. These infection-associated and non-infection-associated factors can lead to a state of chronic inflammation of the liver [4]. Over time, the chronic inflammatory microenvironment may gradually and imperceptibly promote the development of liver fibrosis and early liver cancer, as well as the development, invasion and metastasis of tumor cells.

The article "Relationship between epithelial-to-mesenchymal transition and the inflammatory microenvironment of hepatocellular carcinoma" was published in 2018. Journal: J Exp Clin Cancer Res.

Biological behaviors, such as early invasion, metastasis and recurrence, are challenges to the clinical treatment of liver cancer. Specifically, EMT is considered to be a key step for tumor invasion and metastasis [5]. Tumor cells develop powerful invasive and metastatic ability through the EMT process, which allows the migration of tumor cells to different sites via the circulatory system [6]. In HCC, the long-term chronic inflammatory microenvironment is undoubtedly the decisive factor in the development of the tumor. Inflammatory cell aggregation, inflammatory cell infiltration and inflammatory mediator-induced activation of related pathways are critically involved in tumor invasion and metastasis. However, the association between the occurrence of EMT and the inflammatory microenvironment in the tumor is not yet clear. Here, we review the current knowledge regarding this issue.

### The inflammatory microenvironment of hepatocellular carcinoma

HCC is a typical inflammation-related tumor. The process of tumor growth and infiltration is always accompanied by apoptosis or necrosis, which causes the release of numerous inflammatory mediators. Tumor cells and inflammatory cells also produce chemokines, cytokines, and growth factors, which induce angiogenesis and further inflammation [7]. These inflammatory mediators, inflammatory cells and tumor cells interact to form an inflammatory cascade reaction. Moreover, the persistent inflammatory microenvironment not only promotes tumor induction, but also accelerates tumor progression and promotes the formation of new blood vessels [8], activation of cancer-associated fibroblasts (CAF) [9] and remodeling of the extracellular matrix (ECM) [10]. These conditions also enhance tumor cell survival and proliferation, which play a significant role in the occurrence, development and metastasis of tumors.

### Epithelial-to-mesenchymal transition

Recent studies have shown that EMT is a key step in tumor invasion and metastasis [5, 11, 12]. Normal epithelial cells are highly ordered and have close intercellular connections. These cells also exhibit significant polarity of the free and basal surfaces, with relatively stable morphology. In contrast, interstitial cells, which assist the parenchymal cells to perform organ functions, have different forms and a loose arrangement [13]. They typically lack polarity and have greater migration and invasive capacity. EMT refers to the disruption of tight intercellular junctions among epithelial cells under specific conditions, resulting in loss of the original polarity, order and consistency. Under these circumstances, epithelial cells tend to show interstitial cell characteristics and develop the capacity for migration and apoptosis is inhibited [14].

The article "Relationship between epithelial-to-mesenchymal transition and the inflammatory microenvironment of hepatocellular carcinoma" was published in 2018. Journal: J Exp Clin Cancer Res.

### The molecular mechanism of epithelial-to-mesenchymal transition

The most significant feature of the surface of a cell following EMT is the decrease in E-cadherin expression and the increase in N-cadherin expression [15]. E-cadherin is a connecting structure among epithelial cells and has strong and stable adhesion properties. N-cadherin, which can be defined as the connecting structure among mesenchymal cells, shows weaker adhesion ability, a characteristic that is one of the causes underlying the increase in cell migration and invasion following EMT [16]. The dynamic properties of the intermediate filament protein vimentin are very important for cell flexibility and increased expression of vimentin is an important sign of EMT in tumor invasion and metastasis [17].

The common transcription factors Snail, Slug, Twist, ZEB1, ZEB2, FOXC1, and FOXC2 participate in the induction of the EMT process [18] by reducing E-cadherin expression via intracellular signaling pathways, such as the JAK/STAT3, MAPK/ERK, and PI3K/AKT [19–21]. In addition, many growth factors, such as epidermal growth factor (EGF), transforming growth factor-beta (TGF-β) and platelet-derived growth factor (PDGF), also play a role in the intracellular conduction pathway [17, 22, 23].

### The relationship between the inflammatory microenvironment of hepatocellular carcinoma and the epithelial-to-mesenchymal transition process

The occurrence and development of HCC are accompanied by a persistent inflammatory reaction. Inflammatory cells, inflammatory mediators, and the products of the infecting virus have a great influence on the process of EMT in hepatocellular carcinoma.

### Inflammatory cells in the inflammatory microenvironment of hepatocellular carcinoma

Similar to other tumor microenvironments, inflammatory cells in the HCC microenvironment include mainly macrophages, neutrophils, lymphocytes, mast cells, dendritic cells, and eosinophils. Among these tumor-related macrophages, infiltrating lymphocytes and neutrophils are the three most common leukocytes [24].

#### Tumor-associated macrophages (TAMs) and EMT in hepatocellular carcinoma

Tumor-related macrophages are the primary inflammatory cells infiltrating in the tumor microenvironment [25]. These cells, which have a high degree of heterogeneity and plasticity and are derived from circulating monocytes and Kupffer cells, are recruited into tumor tissues by chemokines, vascular endothelial growth factor (VEGF) and macrophage colony-stimulating factor (MC-SF). Under the influence of cytokines and microbial products, TAMs show specific features of specialization and polarization [24, 26].

The article "Relationship between epithelial-to-mesenchymal transition and the inflammatory microenvironment of hepatocellular carcinoma" was published in 2018. Journal: J Exp Clin Cancer Res.

According to the characteristics of polarization, macrophages can be divided into M1 and M2 subtypes. In the tumor microenvironment, the M2 phenotype tends to predominate, which promotes tumor invasion and metastasis [27]. TAMs are not intrinsically malignant. Nevertheless, their interactions with tumor cells can directly promote tumor growth, invasion and metastasis, and their association with EMT can also be mediated by secreting inflammatory factors, cytokines and related proteases.

In HCC, TAMs are the major cell type promoting tumor invasion and metastasis [7, 25, 28] and their secreted inflammatory cytokines as well as other cytokines and proteases are the main mediators that promote EMT. TAMs induce EMT of tumor cells by secreting factors such as interleukelin-6 (IL-6), interleukelin-8 (IL-8), tumor necrosis factorα (TNFα), TGFβ, EGF, VEGF, matrix metalloproteinase-2 (MMP-2) and MMP-9. Additionally, these factors act synergistically to stimulate neovascularization, degrade the matrix and promote local invasion and distant metastasis of tumor cells (Fig. 1).

**Fig. 1:** Tumor-associated macrophages and epithelial-to-mesenchymal transition in hepatocellular carcinoma. TNFα binds to the receptor TNFR (mainly TNFR1) to phosphorylate PKD2, which then forms a complex with PI3K. This complex stabilizes the high expression of β-catenin via the PI3K/AKT/GSK-3β pathway, upregulates Snail and Twist transcription, and participates in the process of epithelial-to-mesenchymal transition (EMT) to promote tumor invasion and metastasis. IL-8 secreted by TAMs participates in the EMT via the JAK2/STAT3/Snail pathway. It also activates FOXC1 via PI3K/AKT HIF-1α, leading to transactivation of CXC chemokine receptor (CXCR) and CC chemokine ligand 2 (CCL2), otherwise, neurotensin (NTS) and IL-8 are also activated abnormally, leading to upregulated expression of VEGF and MMP9 via the NTS/IL-8 pathway. IL-6 induces EMT by binding to the IL-6R receptor to induce STAT3 phosphorylation via the JAK/STAT3 pathway, leading to downregulated E-cadherin expression and upregulated vimentin expression. This interaction can also induce upregulation of the expression of Snail, ZEB1, ZEB2, Twist and other transcription factors to promote tumor metastasis. TGFβ secreted by TAMs modulates the expression of EMT-related genes at the epigenetic level via the classic TGF-β/TGF-β R/Smad signaling pathway. It also acts on Snail, Slug and other transcription factors via the RhoA/Cdc42, JKN/p38, Erk1/2 and PI3K/Akt pathways. EGF binds to hepatoma cell epidermal growth factor receptor (EGFR), activating downstream ERK/PI3K/AKT, ras/raf/MEK/MAPK, NF-κB and other pathways

IL-6 secreted by TAMs is an important factor involved in the occurrence and development of tumors [29, 30]. It is relatively clear that IL-6 mediates EMT mainly via the IL-6/STAT3 pathway. In this process, IL-6 binds to its receptor IL-6R, which consists of two polypeptide chains; a ligand-binding chain (GP80) and a signal conduction chain (GP130). The latter is phosphorylated following interaction with Janus kinase resulting in activation of STAT3 to form two homologous polymers that enter the nucleus to regulate transcription and promote EMT, a process that is observed in liver cancer [31]. Studies in both human samples and human HCC cell lines in vitro have shown that the IL-6/STAT3 axis comprises a variety of “circuits”, including microRNAs such as miR-24, miR-629, and miR-124, and hepatocyte nuclear factor 4α (HNF4α). In this circuit, IL-6/STAT3 activates the transcription of miRNAs, such as miR-24 and miR-629, which inhibit the activity of HNF4α. HNF4α is an important factor in the maintenance of the growth and normal biological functions of hepatocytes. When its activity is inhibited, hepatocytes enter the inflammatory state, which is exacerbated via a positive feedback mechanism resulting in a severe inflammatory microenvironment that promotes tumor invasion and metastasis (Fig. 2). That is quite similar to the “snowball effect”, with miR-124 representing the key factor in this circuit. In HepG2 and SNU-449 cells, it has been shown that miR-124 suppresses STAT3 activation, restores the function of HNF4α and terminates the further development of the inflammatory environment. Furthermore, miR-124 was shown to inhibit the tumor invasion and metastasis in a mouse model [32]. The effectiveness of this approach has also been confirmed in studies of lung adenocarcinoma, breast cancer and head and neck tumors [33]. In addition to activating the JAK/STAT3 pathway via phosphorylation of STAT3, the IL-6/IL-6R interaction leads to low E-cadherin expression and high vimentin expression as well as upregulated expression of Snail, ZEB1, ZEB2, Twist and other transcription factors that promote tumor metastasis [34–36].

The article "Relationship between epithelial-to-mesenchymal transition and the inflammatory microenvironment of hepatocellular carcinoma" was published in 2018. Journal: J Exp Clin Cancer Res.

**Fig. 2:** HNF4α feedback circuit in hepatocellular oncogenesis. IL-6/STAT3 activates the transcription of miRNAs, such as miR-24 and miR-629, which inhibit the activity of HNF4α. HNF4a directly regulates miR-124 expression. MiR-124 can suppresses STAT3 activation, restores the function of HNF4α. When IL-6/STAT3 pathway is activated, HNF4α activity is inhibited, miR-124 levels is reduced, hepatocytes enter the inflammatory state, which is exacerbated via a positive feedback mechanism resulting in a severe inflammatory microenvironment that promotes tumor invasion and metastasis

IL-8 is another important inflammatory factor secreted by TAMs in HCC. Its expression is associated with tumor growth and survival, as well as increased tumor invasion, migration and angiogenesis. Studies in MHCC97H and HepG2 cell lines have shown that the IL-8 secreted by TAMs participates in EMT via the JAK2/STAT3/Snail pathway [37]. Studies in both human HCC cell lines and mouse models have shown that IL-8 also activates FOXC1 via PI3K/AKT HIF-1α to promote the invasion and metastasis of HCC by trans-activation of CXC chemokine receptor (CXCR) and CC chemokine ligand 2 (CCL2) [38]. The increased IL-8 levels also lead to a higher incidence of portal vein invasion [39]. During the development of HCC, the neurotensin (NTS)/IL-8 signaling pathway is also activated abnormally, leading to increased expression of VEGF and MMP9. These factors co-mediate the process of tumor EMT to promote tumor invasion and metastasis, which has an adverse effect on prognosis [40]. Furthermore, the role of IL-8 in EMT has also been confirmed in pancreatic, breast, prostate and ovarian cancer [41–43].

TNFα is another important inflammatory factor secreted by TAMs in HCC [44]. Studies in human HCC cell lines and mouse models showed that the expression of TNFα and protein kinase D2 (PKD2) in the metastatic liver cancer tissues are significantly higher than that in normal tissues [45]. Moreover, binding of TNFα to the receptor TNFR (mainly TNFR1) on the cell membrane surface induces phosphorylation of intracellular PKD2, which then forms a complex with PI3K to stabilize the high expression of β-catenin via the PI3K/AKT/GSK-3β pathway and participate in EMT to promote tumor invasion and metastasis. The role of TNFα has also been confirmed in other tissues, including malignant tumors, such as tongue cancer, laryngeal carcinoma, cholangiocarcinoma, thyroid cancer and colorectal cancer. Nonetheless, the mechanisms underlying the influence of TNFα are varied, and include the promotion of stromal cell-derived factor-1 (SDF1) secretion in the tongue cancer, high expression of the Snail gene in cholangiocarcinoma and colorectal cancer, and upregulation of Twist transcription in laryngeal carcinoma [46–51].

The TGFβ secreted by TAMs changes the expression of EMT-related genes at the epigenetic level via the classic TGF-β/TGF-βR/Smad signaling pathway [52, 54]. In a study of HCC, Reichl et al. [53] showed that TGFβ-overexpression inhibited the Smad pathway but not the EMT process. TGFβ can also act on Snail, Slug and other transcription factors via the RhoA/Cdc42, JKN/p38, Erk1/2 and PI3K/Akt pathways to downregulate E-cadherin expression and upregulate vimentin expression and mediate EMT in tumor cells [54–56].

The article "Relationship between epithelial-to-mesenchymal transition and the inflammatory microenvironment of hepatocellular carcinoma" was published in 2018. Journal: J Exp Clin Cancer Res.

TAMs can also produce EGF, which binds to hepatoma cell epidermal growth factor receptor (EGFR) to activate downstream signaling pathways, including the ERK/PI3K/AKT, ras/raf/MEK/MAPK, and NF-κB pathways. As a result, EGF downregulates E-cadherin and upregulates vimentin to induce EMT by activation of STAT3 [57–59]. Similarly, it has also been confirmed that VEGF induces EMT in the highly metastatic hepatoma cell line MHCC97H [60]. Finally, members of the MMP family, including MMP-1, MMP-2, MMP-7 and MMP-14, also play an important role in the EMT process in liver cancer [61–63]. In addition, MMP-8 also mediates positive feedback regulation of TGFβ, and participates in the process of EMT via the downstream PI3K/Akt/Rac1 pathway [64].

In conclusion, TAMs are one of the most important inflammatory cell types in the inflammatory microenvironment of HCC. These cells secrete numerous inflammatory factors, which are significant in the EMT process in HCC.

#### Tumor-associated neutrophils (TANs) and HCC EMT

In the occurrence and development of HCC, tumor-associated neutrophils (TANs) also play an important role. Similar to TAMs, TANs also differentiate into two phenotypes; N1 and N2. The N1 phenotype inhibits tumor growth, while N2 promotes tumor growth and metastasis [65]. Specifically, N2 type TANs secrete a variety of cytokines, such as CCL2, neutrophil elastase (NE), hepatocyte growth factor (HGF), MMP9, and VEGF, which affect the growth, angiogenesis, invasion and metastasis of the tumor [66–69] (Fig. 3).

**Fig. 3:** Tumor-associated neutrophils (TANs) and epithelial-to-mesenchymal transition in hepatocellular carcinoma. CCL2 secreted by TANs associates with IL-8 to promote epithelial-to-mesenchymal transition (EMT) via the PI3K/AKT HIF-1α pathway. TANs also upregulate the downstream ZEB1 transcription factors by secreting NE. In addition, HGF promotes EMT of tumor cells and increases hematogenous dissemination by binding to its receptor c-Met. In the absence of p53 gene expression, HGF/Met also mediates EMT of hepatocellular carcinoma by upregulation of Snail and other transcription factors

In a study of human HCC cell lines and mouse models, Huang et al. [38], found that TANs secrete large amounts of CCL2, which interacted with IL-8 to participate in EMT, and reduce the therapeutic effect of sorafenib [70]. Zhou et al. [71] verified these findings in a study of tissue specimens from 452 patients. CCL2, which is a member of the chemotactic factor family, is a low molecular weight protein responsible for leukocyte migration to sites of infection. Moreover, CCL2 interacts with Snail factors in EMT of pancreatic cancer cell lines, melanoma cells and colon cancer cell lines in vitro [72]. CCL2/CCR2 also cooperates with IL-6 to activate the STAT3-Twist pathway in EMT of non-small cell lung cancer [34].

The article "Relationship between epithelial-to-mesenchymal transition and the inflammatory microenvironment of hepatocellular carcinoma" was published in 2018. Journal: J Exp Clin Cancer Res.

NE, which is another important inflammatory mediator secreted by TANs, participates in the invasion and development of lung, ovarian and pancreatic cancer as well as the EMT [73–75]. A study of the Huh7 HCC cell line and 115 patient HCC tissue samples indicated that, during tumor progression, TANs upregulate the downstream ZEB1 transcription factors by secreting NE. It also reduces the expression of cytokeratin and E-cadherin and increases the expression of beta-catenin to mediate the EMT of hepatoma cells [75].

HGF is also one of the cytokines secreted by TANs [76]. By constructing the circulating tumor cell model of liver cancer in mice, Olorunseun et al. [77] showed that HGF promotes EMT of tumor cells and increases hematogenous dissemination by binding to its receptor c-Met. Liu et al. [78] also confirmed that in the absence of the p53 gene, HGF/Met mediates EMT of HCC by upregulation of Snail and other transcription factors. The role of HGF in promoting EMT has also been confirmed in non-small cell lung cancer, prostate cancer and others [79, 80].

The role of MMPs and VEGF in EMT has been described previously. In different tissues, these two factors are secreted by different cells, although their functions are similar.

In conclusion, the essential role of TANs in EMT of HCC is mediated by cytokines, such as NE, HGF and CCL2.

#### Tumor-infiltrating lymphocytes and EMT of HCC

Tumor-infiltrating lymphocytes (TILs) were first discovered and reported by the Rosenberg group in 1986 [81–83]. The level of infiltration is closely related to the prognosis of HCC. Among the TILs, Treg cells (CD4+ CD25+ FoxP3+) are most closely related to the occurrence and development of tumors. Treg cells weaken the function of CD8 + T cells and inhibit the effects of cytotoxic CD8 + T cells on malignant tumor cells, thus, promoting the development of HCC. In HCC patients, high levels of Treg cells in pre-operative circulating blood are closely related to high mortality and low survival rates. Therefore, the imbalance between Treg cells and cytotoxic T cells can be used as a prognostic factor for HCC patients [84, 85].

The article "Relationship between epithelial-to-mesenchymal transition and the inflammatory microenvironment of hepatocellular carcinoma" was published in 2018. Journal: J Exp Clin Cancer Res.

There are few reports of the role of Treg cells in EMT in HCC. However, in study of the breast cancer cell lines BT474 and MCF-7 [86], Treg cells were shown to activate the downstream Smad signaling pathway via the TGFβ pathway, which promoted EMT of breast cancer cells, increased the local frequency of cancer stem cell (CSC)-like cells, and enhanced their invasion and migration ability.

### Inflammatory mediators in the microenvironment of HCC

In addition to the influence of inflammatory cells on the EMT of HCC, various kinds of inflammatory factors also participate in the EMT process of HCC, either directly or indirectly (Fig. 4).

**Fig. 4:** Inflammatory mediators in the microenvironment of hepatocellular carcinoma. HIF-1α promotes vasculogenic mimicry (VM) and epithelial-to-mesenchymal transition (EMT) by upregulation of LOXL2. HIF-1β downregulates E-cadherin expression via the Notch signaling pathway, and interacts with numerous oncogene-encoded proteins including epidermal growth factor receptor (EGFR), c-Myc, K-Ras, even some lncRNAs, such as NEAT1, to promote EMT. CXCL1 participates in tumor promotion by stimulating mitochondrial metabolism and activating EMT. CXCL10 upregulates MMP-2 expression to participate in EMT; MMP-16 and MMP-9 are also key factors. cPLA2 plays an opposing role in TGF-β-induced signaling pathways by inhibiting Smad2/3 phosphorylation and promoting activation of PI3K/AKT/ERK signaling pathways to mediate EMT. PD-1/PD-L1 induces EMT via the PI3K/AKT and ERK/MEK signaling pathways, and upregulation of SREBP-1c

Hypoxia inducible factor (HIFs), which are also involved in tumor inflammation, enhance the metabolic activity of the tissue by causing infiltration of inflammatory cells and inflammatory reactions. The resulting increase in inflammation and the associated inflammatory reaction leads to the increased demand for oxygen. The inflammatory factors also cause vasoconstriction, which further reduces oxygen levels in the inflammatory environment. As a result, high levels of HIFs are generated in the hypoxic microenvironment [87].

HIF-1 (HIF-1α and HIF-1β) is the most common HIF expressed during the development of HCC, which is associated with long-term chronic inflammation. Studies have shown that HIF-1α in the inflammatory microenvironment of HCC promotes vasculogenic mimicry (VM) and the occurrence of EMT by upregulation of LOXL2 [88]. HIF-1β is involved in the EMT process by downregulation of E-cadherin expression via the Notch signaling pathway [89]. HIF-2α interacts with many oncogene-encoded proteins, including EGFR, c-Myc and K-Ras, which participate in the tumor development. HIF-2α also promotes EMT in HCC through upregulation of the lncRNA NEAT1 [90, 91].

The article "Relationship between epithelial-to-mesenchymal transition and the inflammatory microenvironment of hepatocellular carcinoma" was published in 2018. Journal: J Exp Clin Cancer Res.

Similar to the previously mentioned CC chemokine family, the CXC chemokine family, especially CXCL1 and CXCL10, also plays an important role EMT in HCC. CXCL1 promotes tumorigenesis by stimulating mitochondrial metabolism and activating the EMT process [92]. CXCL10 is involved in EMT by upregulating MMP-2 expression [93], and similarly, MMP-16 and other MMPs are also key factors in EMT [94].

T cell immunoglobulin mucin-3 (Tim3) is a specific target for activating T cells in inflammatory responses [95]. In the SMMC-7721 cell line, Tim-3 overexpression upregulated the expression of Snail, Slug, Twist 1, MMP-9 and other transcription factors and enhanced the EMT process compared with that observed in the control group [96].

cPLA2 is one a member of the phospholipase family, the main physiological function of which is to reconstruct the phospholipid structure and to promote the autogenous removal of necrotic tissue. Inflammation can be mediated by COX-1 (cyclooxygenase − 1), releases arachidonic acid through oxidation and peroxide, and leads to the biosynthesis of prostaglandins, especially prostacyclin, which induce inflammation and pain [97]. Using a xenograft tumor transplant model, Fu et al. [98] showed that cPLA2 can play an opposing role in TGF-β-induced signaling pathways by inhibiting Smad2/3 phosphorylation and promoting the activation of PI3K/AKT/ERK pathways to mediate EMT of HCC.

Programmed cell death receptor-1 (PD-L1) is a transmembrane receptor present on T cells. It was first identified in an apoptotic T cell hybridoma and named based on its involvement in apoptosis [99]. Although PD-1/PD-L1 is not an inflammatory factor, it is widely expressed in the liver tissues of patients with chronic HBV infection and even liver cancer [100, 101]. Additionally, in patients with a more aggressive HCC and shorter survival, Critella et al. [102] found a markedly immunosuppressed microenvironment (as shown by the local upregulation of both PD-1 and PD-L1) against a background of higher systemic inflammation, with a distinct switch toward EMT and extremely poor differentiation at the histological level compared with the conditions detected in patients with a less aggressive disease and longer survival. However, the specific mechanisms were not investigated. In other studies of the relationship between PD-1/PD-L1 and EMT, Alsuliman et al. [103] showed that PD-L1 induced EMT in tumor cell lines via the PI3K/AKT and ERK/MEK pathways in breast cancer and that the involvement of the PI3K/AKT pathway was more important in this process. Wang et al. [104] found that PD-L1 induced EMT and enhanced RCC cell cancer stemness through upregulation of SREBP-1c in the renal cell carcinoma (RCC) cancer cell lines, 769P and ACHN. Furthermore, the relationship between PD-L1 and EMT has also been recently demonstrated in head and neck squamous cell carcinoma, esophageal cancer, and pulmonary adenocarcinoma [105–107]. PD-1/PD-L1 also plays important roles in regulating T cell proliferation and differentiation and maintaining autoimmune tolerance, as well as the development of tumor immune escape and chronic infection [108].

The article "Relationship between epithelial-to-mesenchymal transition and the inflammatory microenvironment of hepatocellular carcinoma" was published in 2018. Journal: J Exp Clin Cancer Res.

### Virus-related products in the inflammatory tumor microenvironment

The occurrence and development of liver cancer is closely related to hepatitis virus infection, especially HBV and HCV. The products of viral expression are important factors that affect the development, invasion and metastasis of liver cancer (Fig. 5).

**Fig. 5:** Virus-related products in the inflammatory tumor microenvironment. HBx stabilizes the transcription of Snail in the PI3K/AKT/GSK-3b pathway to mediate epithelial-to-mesenchymal transition (EMT). It also participates in the EMT process by inducing upregulation of Twist expression and activation of STAT3 transcription. In addition, HBx activates c-Src and mediates the expression of IGF2 in the SUMO pathway, or directly upregulates the expression of bHLH transcription factor E12/E47, which inhibits E-cadherin expression and induce EMT. NS3 promotes EMT by downregulating PPM1A through ubiquitination. It also enhances cancer cell invasion by activating matrix metalloproteinase-9 (MMP-9) and cyclooxygenase-2 (COX-2) via the ERK/p38/NF-κB signaling cascade, and interacts with p53 to inhibit p53-dependent transcription. NS4B upregulates the Snail transcription factor via the PI3K/AKT signaling pathway and induce EMT

In China and Africa, most patients with HCC are infected with HBV. The HBV genome mainly includes four overlapping open reading frames (ORFs): S, C, P and X. The S ORF is divided into PreS1, PreS2 and S, which are translated predominantly into virus surface antigen or virus envelope protein. The C ORF contains two intra-frame codons, encoding HBV core protein (HBc) and HBV e antigen (HBe), respectively. The P ORF encodes a DNA polymerase protein, which also has reverse transcriptase activity and is responsible for replication of the HBV genomic DNA. The X ORF encodes the X protein, which is considered to be the key factor in the occurrence and progression of liver cancer. It has a wide range of non-specific transactivation effects and functions. In the nucleus, HBx cannot directly bind the double-stranded DNA, but it can combine with the transcription factors through protein-protein interactions. HBx also mediates the formation of the transcriptional initiation complex and participates in the EMT process of HCC [109]. In studies of the Huh-7 and SMMC7721 cell lines, Liu and Lu et al. [110, 111] showed that HBx stabilizes the transcription of Snail, including its superfamily member Snail1, to mediate EMT via the PI3K/AKT/GSK-3β signaling pathway. Teng et al. [112] also showed that HBx is involved in the upregulation of Twist expression and activation of STAT3 transcription leading to EMT in the MHCC97H and HL-7702 cell lines. In addition, HBx has been shown to activate c-Src (a non-receptor tyrosine kinase) to induce the expression of insulin-like growth factor 2 (IGF2), and reduce E-cadherin expression via the small ubiquitin like small ubiquitin-related modifier (SUMO) pathway to induce EMT in the SMMC-7721 hepatoma cell line [113, 114]. A study of the HepG2 and HUH-7 cell lines also suggested that HBx directly upregulates expression of the bHLH transcription factor E12/E47, inhibits E-cadherin expression, and induces the process of EMT [115, 116]. In contrast, Wang et al. [117] demonstrated that EMT was suppressed in the HepG2.2.15 cell line in the presence of high levels of HBV virus replication. However, the underlying mechanism is still unclear, and moreover, the effect of virus on EMT in liver cancer may not be dependent only on HBx levels, an issue which requires further investigation.

The article "Relationship between epithelial-to-mesenchymal transition and the inflammatory microenvironment of hepatocellular carcinoma" was published in 2018. Journal: J Exp Clin Cancer Res.

In Europe, America and Japan, HCV infection is the main cause of hepatitis infection. The HCV genome includes 5′-untranslated region, an ORF encoding 3011 amino acids and a 3′-untranslated region. The ORF encodes a large precursor protein, which can be processed to form 10 proteins (structural proteins, core, E1, E2 and P7, and non-structural protein, NS2–5) [118]. Accumulating experimental evidence suggests that HCV contributes to HCC by directly modulating signaling pathways that promote the malignant transformation of hepatocytes [119]. Among the HCV-encoded proteins, the core proteins NS3, NS4B, and NS5A have received much attention, since all of them possess cell-transforming potential by interacting with a number of host factors and signaling pathways when expressed in cell culture or transgenic animal models [120]. Zhou et al. [121] found that NS3 promotes EMT in the Huh-7 and Huh-7.5.1 cell lines by inducing the decomposition and downregulation of protein phosphatase 1A (PPM1A) through ubiquitination. In addition, Lu et al. [122] suggested that in the HepG2 and Huh7.5.1 cell lines, NS3 also enhances cancer cell invasion by activating MMP-9 and COX-2 via the ERK/p38/NF-κB signal cascade, and interacts with p53 to inhibit p53-dependent transcription [123]. In the same way, NS4B also increases expression of the Snail transcription factor via the PI3K/AKT pathway and induces EMT in liver cancer [124].

The article "Relationship between epithelial-to-mesenchymal transition and the inflammatory microenvironment of hepatocellular carcinoma" was published in 2018. Journal: J Exp Clin Cancer Res.

## Conclusions

The importance of EMT in the invasion and metastasis of HCC has gradually been clarified. There is no doubt that the inflammatory microenvironment formed by the inflammation associated with hepatitis virus infection is an important factor affecting the invasion and metastasis of liver cancer. The virus not only participates in the process of liver inflammation, but also directly promotes the development of the tumor by combining with the host genome and encoding proteins. However, numerous transcriptional factors are involved in EMT, and many pathways are activated by inflammatory factors. The cytokines involved in the inflammatory microenvironment are also complex. Although knockout or overexpression of relevant genes has been shown to block tumor invasiveness metastasis in cells and small animal models, this strategy is still far from clinical application. On the one hand, despite blocking an individual pathway or inhibiting a single gene, the upstream factors still have many other mechanisms through which to continue to promote tumor progression. On the other hand, the level of gene suppression that can be achieved in cells and small animal models is difficult to apply to large animals or even in the clinic. Furthermore, the cost and prolonged timeframe of research on targeted inhibitory drugs for the identified gene will delay confirmation of the actual clinical effect of the gene modification.

Therefore, the future direction of research will involve investigation of potential commonality among different inflammatory factors in promoting the EMT of HCC, as well as strategies to modulate the tumor microenvironment or block the expression of inflammatory factors and signaling pathways to inhibit EMT. We anticipate that control of hepatitis will play a decisive role in the treatment of inflammatory-related tumors like HCC. Similar to TNF, TGF, EGF, IL-8, PLA2 and other inflammatory factors, the virus-encoded proteins HBx and NS3, NS4B also signal via classic conduction pathways such as PI3K/AKT/GSK3β and ERK/NF-κB. This may account for the interaction of viral gene-coding proteins and inflammatory factors produced in the microenvironment. Elimination of viral infection and control of inflammatory responses may be an important approach to inhibiting tumor progression, invasion and metastasis in the future.

## Abbreviations

CCL2: CC chemokine ligand 2
CSCs: Cancer stem cells
CXCR: CXC chemokine receptor
EGF: Epidermal growth factor
EGFR: Epidermal growth factor receptor
EMT: Epithelial-to-mesenchymal transition
HBV: Hepatitis B virus
HCC: Hepatocellular carcinoma
HCV: Hepatitis C virus
HGF: Hepatocyte growth factor
HIFs: Hypoxia inducible factor
HNF4α: Hepatocyte nuclear factor 4α
IL-6: Interleukelin-6
IL-8: Interleukelin-8
MET: Mesenchymal-epithelial transition
MMP-2: Matrix metalloproteinase-2
MMP-9: Matrix metalloproteinase-9
NTS: Neurotensin
PDGF: Platelet-derived growth factor
PKD2: Protein kinase D2
SDF1: Stromal cell-derived factor-1
TAMs: Tumor related macrophages
TANs: Tumor Related Neutrophils
TGF-β: Transforming growth factor factor
Tim3: T cell immunoglobulin mucin-3
TNFα: Tumor necrosis factorα
VEGF: Vascular endothelial growth factor
VM: Vasculogenic mimicry
COX-1: (cyclooxygenase − 1)
PD-1: Programmed cell death receptor-1
HBc: HBV core protein
HBe: HBV e antigen
IGF2: Insulin-like growth factor 2
SUMO: Small ubiquitin-related modifier
ORF: Open reading frame
PPM1A: Protein phosphatase 1A
MMP-9: Matrix metalloproteinase-9
COX-2: Cyclooxygenase-2
